# Foreign Direct Investment, Regional Innovation, and Green Economic Efficiency: An Empirical Test Based on the Investigation of Intermediary Effect and Threshold Effect

This article has been retracted.

**DOI:** 10.1155/2021/7348599

**Published:** 2021-09-30

**Authors:** You-Qun Wu, Huai-Xin Lu, Xin-Lin Liao, Jia-Bao Liu, Jia-Ming Zhu

**Affiliations:** ^1^School of Economics, Anhui University of Finance and Economics, Bengbu 233030, Anhui, China; ^2^School of Mathematics and Physics, Anhui Jianzhu University, Hefei 230601, China; ^3^Institute of Quantitative Economics, Anhui University of Finance and Economics, Bengbu 233030, China

## Abstract

Based on the theoretical mechanism analysis of FDI, regional innovation, and green economic efficiency, this article uses China's provincial panel data to calculate the provincial green economic efficiency level based on the three-stage DEA method and uses the system GMM model, intermediary effect model, and threshold model to empirically test the specific effects and transmission paths of FDI on the efficiency of the green economy. Research shows that FDI is one of the important factors that promote the improvement of green economic efficiency. Subregional tests have found that FDI has a significant regional heterogeneity in promoting the efficiency of the green economy. The mediation effect test found that the mediation effect of regional innovation is significant, and FDI can significantly promote the growth of green economic efficiency through regional innovation. The threshold effect analysis found that there are significant and effective double thresholds for regional economic levels, and the impact of FDI on green economic efficiency is heterogeneous within different threshold intervals. The research conclusions provide new inspiration for China to allocate FDI more rationally and efficiently under the new development pattern.

## 1. Introduction

Since the reform and opening up, China's “Special Management Measures for Foreign Investment Access (Negative List)” project has continued to reduce, and the “Notice on Several Measures to Actively and Effectively Use Foreign Investment to Promote High-quality Economic Development” has continued to expand the scope of opening up. In 2020, China absorbed total foreign investment to US $163.9 billion, up by 4% from the previous year, accounting for 19% of the global foreign direct investment (Foreign Direct Investment, FDI), realizing the “three increases” in the total investment volume, the growth range, and the global proportion. In the new development stage, China's development environment is facing profound and complex changes. The 14th five year plan and the outline of long-term objectives for 2035 run through a clear main line; that is, we should unswervingly implement the new development concept and list “implementing high-level opening to the outside world and promoting the stability and quality improvement of foreign trade and foreign investment” as one of the key tasks. One belt, one road to building a high-quality economy and the need to participate in global economic governance reform and improvement, is the foundation for opening up a new economic system at a higher level. As an important way of international high-tech technology spillover, FDI can promote the reverse spillover of high-tech developing countries and has a significant impact on the industrial structure, unemployment rate, and productivity of the host country [1]. At present, China is in the context of “double cycle,” and the government needs to optimize the level and structure of foreign capital and comprehensively enhance the integration of foreign capital and local economy [2]. What is the impact of FDI and regional innovation on green economic efficiency? What is the impact of FDI on green economic efficiency heterogeneous? A series of problems can provide new enlightenment for China's more reasonable and efficient allocation of FDI under the new development pattern.

## 2. Literature Review

The influence of FDI on the host country has been a key area of scholars. Scholars have discussed the impact of FDI on the economic growth, resources, and environment of the host country from different perspectives, mainly with the following views: (1) FDI can significantly promote the economic growth of the host country. Some scholars believe that the most direct effect of FDI on the host country is the accumulation effect of material capital, and the lack of financial support in the early stage of economic development leads to the obstruction of regional development. The introduction of FDI can provide capital for the infrastructure construction of the host country, improve the capital utilization rate, and facilitate the industrial structure upgrading [3]. Second, FDI is the main channel for the cross-border flow of high and new technology. It can promote the improvement of personnel factors through technology spillover effect and industry correlation effect, make up for the lack of personnel factors in host countries [4], and significantly improve the total factor productivity of host countries [5]. (2) The FDI is not conducive to the economic growth of the host country. Relevant studies believe that the large influx of FDI is one of the reasons for the negative economic growth of the host country, which is due to the competition and substitution effects between FDI and the domestic capital of the host country. Initially, the introduction of FDI in the host country will increase its total capital amount, when the continuous increase of FDI will cause its substitution effect and crowding effect gradually significant, making the total domestic capital tends to decline, eventually resulting in the host country capital contraction [6]. There is also a threshold value for the FDI own scale. The FDI scale is less than the threshold value, and the positive effect on the innovation efficiency when it exceeds the threshold value is not significant or even has a negative impact [7]. For developing countries, excessive reliance on FDI, in the early stage of economic development, leads to urbanization attached to the industrialization process, resulting in lag or excessive urbanization [8]. Second, the technical spillover effect of FDI is not idealized for the input host country. The main reason is that it is difficult for the employees of domestic enterprises in the host country to accept the advanced technology and management experience of foreign enterprises. In recent years, foreign-owned enterprises in sole proprietorship or holding form have increased restrictions on technology spillover, reducing the marginal contribution of FDI to economic growth [9]. The spillover effect of FDI is also limited by the host country's own policy environment, economic development level, human capital level, and other factors. When the policy environment is conducive to the introduction of foreign investment and the high level of economic development, the positive spillover effect of foreign investment will be strong. Third, as the host country attaches great importance to high-tech research and development, it promotes the transformation of domestic production technology, so that the technology spillover effect of FDI will be further reduced. Moreover, the technology transfer effect of foreign capital is relatively strong. When the development of foreign capital in the host country is hindered, it will promptly change the investment environment. At this time, the negative effect of FDI will become more significant [10]. Finally, relevant research shows that the industrial correlation effect of FDI does not systematically form a positive spillover of upstream and downstream enterprises but will inhibit the enthusiasm of related enterprises and leads to the vicious competition [11]. (3) Regarding the “Pollution of Heaven” hypothesis, some scholars believe that FDI will aggravate environmental pollution in the host country and exchange “green waters and green mountains” for economic growth. Relevant research shows that, in order for developing countries to solve the problem of lack of capital and technology in the early stage of economic development, they will reduce environmental regulatory standards to attract foreign capital into their own market, resulting in excessive exploitation and utilization of domestic natural resources [12]. The continuous reduction of environmental standards will form the “environmental bottom line competition” phenomenon. The FDI enters the host country without idealized high-tech industry, mostly concentrated on high pollution and high energy consumption industries and forming the occupation of host natural resources, and is not conducive to guide the development of host green industry but intensifies the environmental pollution problem [13]. (4) The “Pollution Aura” hypothesis states that the effects of FDI on technology spillover, industrial correlation, and market competition in the host country will promote the technological progress of the host country, improve the utilization of production factors and reduce pollution emissions, and facilitate the treatment of resource utilization and environmental pollution problems in the host country. The main reason is that developed countries are more stringent standards for waste discharge from enterprises and more perfect environmental regulation standards. So, FDI has more advanced production technology and pollutant treatment technology, which can improve the resource utilization rate and reduce the damage to the environment. In addition, the imitation of domestic enterprises in the host country forms the improvement of the production level and harmless waste treatment technology in the host country. The specific study is as follows: Wang et al. research found that FDI significantly promotes the regional green total factor efficiency by improving the input efficiency of labor and energy [14]. Liu and Zhao started from the three industrial wastes and found that FDI will effectively encourage the treatment of traditional pollutants, especially for sulfur dioxide and industrial wastewater [15]. Huang and Zhou analyzed the Yangtze River Economic Belt and found that FDI can effectively inhibit wastewater discharge and promote the optimization of environmental resources [16].

In conclusion, the existing literature has recognized the economic and environmental impact of FDI and explored it, which has an important inspiration for this paper. This paper finds that there is room for further exploration in the empirical research of FDI and economy and environment, mainly in the following aspects: first, most studies favor the unilateral impact of FDI on economic growth or environmental pollution, ignoring the quality of economic development, and comprehensively considering the economic efficiency and environmental factors, management factors, and statistical noise. Second, most literature use grouping or introduce multiplication model to explore the relationship between FDI and economic growth or environmental pollution. Its subjective factors are large and cannot get a specific threshold. In a few threshold models, such as the Hansen static panel threshold model, the premise is more stringent and did not use the subsequent perfect dynamic panel threshold model for empirical analysis. Third, most literature studies whether there is a threshold for FDI's own scale and considers less whether the influence of FDI produces heterogeneity at different economic development levels.

Therefore, the main contributions of this paper are as follows. First, based on the nonexpected output, in the super SBM-DEA model, the environmental factors, management factors, and statistical noise are considered, using the three-stage DEA to obtain the green economic efficiency value. Second, considering the “inertia” of the economic system, using the dynamic system GMM model not only examines the perspective of FDI but also introduces regional innovation into the category of model research and analyzes the role mechanism of FDI on the green economic efficiency. Third, using the dynamic panel threshold model, the nonlinear influence of FDI on green economic efficiency is discussed for different economic development levels.

## 3. Analysis of the Theoretical Mechanism of FDI, Regional Innovation, and Green Economic Efficiency

Based on the model of Ji et al. [17], this paper constructs a theoretical model of the nonlinear relationship between FDI, regional innovation, and green economic efficiency. First, we assume that the green economic efficiency level of a country or region will be affected by regional innovation, productivity, and other factors under regional innovation without technological innovation. Second, it is assumed that green economic efficiency follows the form of C-D production function:

(1) $$\begin{array}{c} {\text{GECM}}_{it}=A_{it}*IN_{it}^{\alpha }*G_{it}^{\beta }. \end{array}$$

Among them, i represents the region; *t* represents the time; the GECM_*it*_ represents the green economic efficiency of expected output, unexpected output, environmental factors, and statistical noise and random noise; *A*_*it*_ represents other factors that may affect the green economic efficiency; IN_*it*_ represents a regional innovation. The coefficient *α* indicates the relationship between regional innovation intensity and green economic efficiency. When *α* > 0 indicates a positive correlation between the two, the stronger the regional innovation, the higher the actual green economic efficiency level. When *α* < 0, there is a negative correlation between the two. When *α* = 0, this indicates that regional innovation is not green economic efficiency. *G*_*it*_ is the efficiency in the production process without considering regional innovation, and its value is mainly determined by the market behavior of enterprise departments in economic activities. The coefficient *β* shows the production department for the productivity of the importance. The value range is 0 < *β* ≤ 1. *β* value means the enterprise of the implementation of innovation research and development productivity. The greater *β* value shows the enterprise innovation research and development productivity attention, and its innovation and development consciousness is weak.

*G*_*it*_ is closely related to *Y*_*it*_, the output of enterprise departments, whether from the perspective of production process or output results, and represents production efficiency. It is related to *H*_*it*_, the technology input in enterprise production process; that is, *G*_*it*_ is related to *H*_*it*_. Thus, the production efficiency *G*_*it*_ is assumed in obedience to the constant alternative elastic production function, and then, *G*_*it*_ can be represented as

(2) $$\begin{array}{c} G_{it}={\left(\gamma_{1}*Y_{it}^{-\rho }+\gamma_{2}*H_{it}^{-\rho }\right)}^{-\left(m/\rho \right)}. \end{array}$$

Among them, 0 < *γ*_1_ ≤ 1; 0 < *γ*_2_ ≤ 1; *ρ* ≥ −1. The introduction of FDI will produce a series of effects such as capital accumulation effects and technology spillover effects, which will directly or indirectly affect *H*_*it*_. Therefore, *H*_*it*_ can be represented by FDI_i*t*_:

(3) $$\begin{array}{c} H_{it}=k*{\text{FDI}}_{it}. \end{array}$$

Among them, *k* > 0. Substituting formulas (2) and (3) into formula (1), we have:

(4) $$\begin{array}{c} {\text{GECM}}_{it}=A_{it}*{\text{IN}}_{it}^{\alpha }*{\left[\gamma_{1}*Y_{it}^{-\rho }+\gamma_{2}*{\left(k*{\text{FDI}}_{it}\right)}^{-\rho }\right]}^{-\left(m\beta /\rho \right)}. \end{array}$$

Then, take the logarithm of (4) as a whole:

(5) $$\begin{array}{c} Ln{\text{GECM}}_{it}=LnA_{it}+\alpha Ln{\text{IN}}_{it}-\frac{m\beta }{\rho }*Ln\left[\gamma_{1}*Y_{it}^{-\rho }+\gamma_{2}*{\left(k*{\text{FDI}}_{it}\right)}^{-\rho }\right]. \end{array}$$

*Ln*[*γ*_1_*∗Y*_*it*_^−*ρ*^+*γ*_2_*∗*(*k∗*FDI_*it*_)^−*ρ*^] in (5) is extended in order 2 at *ρ* = 0:

(6) $$\begin{array}{c} Ln{\text{GECM}}_{it}=LnA_{it}+\frac{m\beta }{\rho }\frac{\gamma_{2}}{\gamma_{1}+\gamma_{2}}Lnk-\frac{m\beta }{\rho }\frac{\gamma_{2}^{2}}{{\left(\gamma_{1}+\gamma_{2}\right)}^{2}}{\left(Lnk\right)}^{2}-\frac{m\beta }{\rho }\frac{\gamma_{2}}{\gamma_{1}+\gamma_{2}}{\left(Lnk\right)}^{2}+\alpha Ln{\text{IN}}_{it}+\frac{m\beta }{\rho }\frac{\gamma_{1}}{\gamma_{1}+\gamma_{2}}\left(1-\frac{2\gamma_{2}}{\gamma_{1}+\gamma_{2}}Lnk\right)*LnY\\ -\frac{m\beta }{\rho }\frac{\gamma_{1}}{\gamma_{1}+\gamma_{2}}\left(1-\frac{\gamma_{1}}{\gamma_{1}+\gamma_{2}}\right)*{\left(LnY\right)}^{2}-\frac{m\beta }{\rho }\frac{\gamma_{2}}{\gamma_{1}+\gamma_{2}}\left(1+\frac{\gamma_{2}}{\gamma_{1}+\gamma_{2}}\right){\left(Ln{\text{FDI}}_{it}\right)}^{2}+\frac{m\beta }{\rho }\frac{\gamma_{2}}{\gamma_{1}+\gamma_{2}}\left(1-Lnk-\frac{2\gamma_{2}}{\gamma_{1}+\gamma_{2}}Lnk\right)*Ln{\text{FDI}}_{it}-\frac{m\beta }{\rho }\frac{2\gamma_{1}\gamma_{2}}{{\left(\gamma_{1}+\gamma_{2}\right)}^{2}}LnY_{it}*Ln{\text{FDI}}_{it}. \end{array}$$

From the previously mentioned formula, FDI has a direct and indirect impact on green economic efficiency, and it is directly affected by *Ln*FDI_*it*_. The coefficient size of the term is reflected. When the coefficient is greater than 0, FDI shows positive effect on the green economic efficiency, and when the coefficient is less than 0, FDI shows negative effect on the green economic efficiency. The LnFDIit presents the square term. When the coefficient is not zero, it indicates that there is a nonlinear variation relation in the role of FDI on the green economic efficiency. The direct impact of regional innovation on green economic efficiency can be expressed by the coefficient *α*.

Based on the analysis of existing literature mechanism, this paper believes that, with the deepening of the global industrial chain division and China's opening policy, China's FDI introduction reached new highs, filled the gap in capital and technology of the economic development, improved domestic innovation and development level, management efficiency, and ecological industrial chain, and promoted the selective flow of capital and labor between enterprises, industries, and regions, reduced enterprise financing constraints and labor difficulties, and realized the improvement of capital allocation efficiency [18]. Moreover, the essence of profit-seeking capital requires that when FDI increases in a certain field, the productivity of related industries in this field will inevitably be improved: promoting the industrial chain capacity upgrading in this field, eliminating backward industries and production capacity, reducing the blind pursuit of capital, waste of environmental resources, and environmental regulation costs, making the high-tech industry favored by domestic and foreign capital, promoting the extensive research and development and application of high-tech in China, and optimizing the market structure [19]. A more reasonably optimized capital labor ratio and the cost of innovation input will significantly promote green technology progress and have a positive effect on green productivity [20]. Based on the previously mentioned analysis, the following assumption is made.
    Hypothesis 1: FDI is conducive to improving the efficiency level of the green economy.
Second, scientific and technological progress is a prerequisite for a country's industrial structure upgrading and sustainable development. A country's development not only depends on the development of its own scientific research and experiment but also needs international exchanges of science and technology. FDI is an important carrier of international science and technology exchanges. The importance of FDI is reflected in not only the rectification of the gap in the host country's capital but also the technology spillover effect, industrial correlation effect, and competition effect on the host country. FDI entering the Chinese market will bring domestic advanced science and technology and management experience. The transnational flow of high-tech will reduce domestic introduction costs and produce technology spillover effect and accelerate the promotion and application of high and new technologies in domestic environmental resources and production capacity [3]. With the industrial correlation effect, when the application of advanced technology is in a link of the industrial chain, the chain adjustments before and after the industrial chain will maintain the technical consistency and stability of the industrial chain and promote the more efficient operation of relevant industries [4]. The competitive effect of FDI also promotes the capital flow. On the one hand, the increase of FDI will squeeze out and replace the inefficient domestic capital and optimize the domestic capital structure. The guiding role of FDI will lead the domestic capital to participate in related industries and enhance the “dry middle school” effect of domestic capital. On the other hand, FDI will enhance the competition among industries, promote industrial capacity upgrading, improve the utilization rate of resources, and be conducive to the improvement of research and development innovation and technological imitation ability [21]. Based on the previously mentioned analysis, the following assumption is made.
    Hypothesis 2: FDI can indirectly affect the green economic efficiency through regional innovation.
Finally, in view of China's reform and opening up, individual cities take the lead in opening up and introducing foreign investment, gradually covering all regions of the country. The economic development level is greatly different in different regions. On the one hand, the level of economic development is the embodiment of the comprehensive strength of industrial structure, financial development level, and science and technology level. There are great differences in preferential policies and business environment attracting foreign investment with different economic development levels. Areas with high level of economic development are more powerful and more attractive to foreign investment. The inclined areas of foreign investors to choose investment will be affected by the level of regional economic development, forming the “path dependence” and further deepening the differences between the capital accumulation effect and technology spillover effect of foreign capital in different regions. On the other hand, regions with higher level of economic development can more efficiently absorb, transform, and utilize FDI capital accumulation effect, technology spillover effect, and a series of effects with higher levels of talents, more perfect industrial chain, higher-tech research, and development capabilities. Based on the previously mentioned analysis, this paper presents the following assumption.
    Hypothesis 3: FDI, at different levels of economic development, has a nonlinear impact on green economic efficiency.

## 4. Model Construction and Variable Description

### 4.1. Research Method

Currently, more scholars use data envelopment analysis (DEA) in productivity studies. Tone proposed a super SBM-DEA model based on relaxation variables for early efficiency measures without considering the effects of relaxation variables and the defects actually used in production activity [22]. Thereafter, Fried and Lovell further considered the impact of environmental factors, statistical noise, and random noise on the efficiency evaluation of DMU and separated them to achieve a more objective and accurate measure [23]. In conclusion, based on the super SBM-DEA model of undesired output, this paper carries out a three-stage processing to measure the efficiency of green economy in China's provinces.

#### 4.1.1. Three-Stage DEA Model

The first stage uses the nonexpected output super SBM-DEA model as the basic model to calculate the initial green economic efficiency value. Assuming that each region is a decision making unit (DMU), for each region the input variable is type *m*, type *T*1 expected output, and type *T*2 nonexpected output, expressed by vectors as *x* ∈ *R*^*m*^, *y*^*g*^*R*^*T*1^, and *y*^*b*^ ∈ *R*^*T*2^. *X*, *Y*^*g*^, and *Y*^*b*^ are defined as matrix: *X* = [*x*_1_,…, *x*_*n*_] ∈ R^*m*^*∗*^*n*^, *Y*^g^ = [*y*_1_^*g*^,…, *y*_*n*_^*g*^] ∈ R^*T*1^*∗*^*n*^, and *Y*^*b*^ = [*y*_*1*_^*b*^,…, *y*_*n*_^*b*^] ∈ *R*^*T*2^*∗*^*n*^. Any element in the matrix is greater than 0. This constructs the collection of environmental technologies, *Q* = {(*x*, *y*^*g*^, *y*^*b*^*) |x* *≥* *Xλ, y*^*b*^ ≥ Y^*b*^*λ, y*^*g*^ ≤ Y^*g*^*λ*, *λ* ≥ 0}. *Q* is a set of production possibilities to measure green economic efficiency, where *λ* is the weight vector. When its sum is 1, the scale remuneration is variable; otherwise, the scale remuneration is unchanged.

Adding the undesired output to the super SBM-DEA model yields a collection of environmental technologies with the following:

(7) $$\begin{array}{c} \bar{Q}=\left\{\left(\bar{x},{\bar{y}}^{g},{\bar{y}}^{b}\right)|\bar{x}\sum_{j=1,\neq 0}^{n}\lambda_{j}x_{j},{\bar{y}}^{b}\geq \sum_{j=1,\neq 0}^{n}\lambda_{j}y_{j}{}^{b},{\bar{y}}^{g}\leq \sum_{j=1,\neq 0}^{n}\lambda_{j}y_{j}{}^{g},y_{j}{}^{g}\geq 0,\;\lambda \geq 0\right\}. \end{array}$$

The super SBM-DEA model considering nonexpected output is shown as follows:

(8) $$\begin{array}{c} \tau^{*}=\text{min}\frac{\left(1/m\right)\sum_{i=1}^{m}\left({\bar{x}}_{i}/X_{i0}\right)}{\left(1/\left(T1+T2\right)\right)\left(\sum_{r=1}^{T1}\left({\bar{y}}_{r}^{g}/y_{r0}^{g}\right)+\sum_{r=1}^{T2}\left({\bar{y}}_{r}^{b}/y_{r0}^{b}\right)\right)}\\ \text{s}.\text{t}.\left\{\begin{array}{c} \bar{x}\geq \sum_{j=1,\neq 0}^{n}\lambda_{j}x_{j},\\ {\bar{y}}^{g}\leq \sum_{j=1,\neq 0}^{n}\lambda_{j}y_{j}^{g},\\ {\bar{y}}^{b}\leq \sum_{j=1,\neq 0}^{n}\lambda_{j}y_{j}^{b},\\ \bar{x}\geq x_{0},\bar{y}\leq y_{0}^{g},{\bar{y}}^{b}\geq y_{0}^{b},\;\lambda \geq 0. \end{array}\right. \end{array}$$

Among them, *λ* is the weight vector and the objective function *τ*^*∗*^ ≥ 1. For a specific evaluated DMU, the larger *τ*^*∗*^ value is, the more efficient the evaluated unit is.

In the second stage, the stochastic frontier model was established, considering the impact of environmental factors, statistical noise, and random noise on green economic efficiency. Based on formula (9), the stochastic frontier model is used to estimate the impact of each environmental variable on the input relaxation variable and test the likelihood ratio. Finally, the input of other DMU is adjusted to the most effective DMU, as shown in formula (10).

(9) $$\begin{array}{c} T_{ni}=f\left(P_{i};\alpha_{n}\right)+\gamma_{ni}+\mu_{ni}. \end{array}$$

Among them, *i* = 1,2,…, *I*; *n* = 1,2,…, *N*. *T*_*ni*_ represents the slack value of the *n*-th input in the *i*-th decision-making unit; *P*_*i*_ is the environment variable, *a*_*n*_ is the environment variable value; *γ*_*ni*_ + *μ*_*ni*_ is the mixed error items, and *γ*ni is the random noise and *μ*ni is statistical noise, which represent the effects of random noise and statistical noise on the input relaxation variables, respectively, where *γ* obeys *N*(0, *σ*^2^) and *μ* obeys *N*^+^(0, *σ*^2^).

(10) $$\begin{array}{c} x_{ni}^{\prime }=x_{ni}+\left\{\text{max}\left[f\left(P_{i};{\hat{\alpha }}_{n}\right)\right]-f\left(P_{i};{\hat{\alpha }}_{n}\right)\right\}+\left[\text{max}\left(\gamma_{ni}\right)-\gamma_{ni}\right]. \end{array}$$

Among them, *i* = 1,2,…, *I*; *n* = 1,2,…, *N*. *x*′_*ni*_ is the adjusted inputs, *x*_*ni*_ is the preadjusted inputs, max [ƒ (P._*i*_; *α*_*n*_*_*_*hat*_)]−ƒ (P_*i*_;*α*_*n*_*_*_*hat*_) is adjusting the environmental factors, and max(*γ*_*ni*_)−*γ*_*ni*_ applies all the decision units to the same condition level.

The third stage replaces the adjusted input variables into the super SBM-DEA model containing nonexpected output, resulting in green economic efficiency values considering environmental factors, random noise, and statistical noise, as shown in Table 1.

#### 4.1.2. Generalized Method of Moments Estimation

The advantage of dynamic system GMM is that it considers the process of dynamic change of variables, increases the horizontal equation participation in estimation, corrects the standard errors of deviation estimator, and improves the accuracy of estimation [21]. The model is built as follows:

(11) $$\begin{array}{c} Ln{\text{GECM}}_{it}=\alpha +\beta_{1}Ln{\text{GECM}}_{it-1}+\beta_{2}Ln{\text{FDI}}_{it}+\beta_{3}Ln{\text{IN}}_{it}+\beta_{4}Ln{\text{SECD}}_{it}+\beta_{5}Ln{\text{RD}}_{it}+\beta_{6}Ln{\text{GGPAY}}_{it}+v_{i}+\varepsilon_{it}. \end{array}$$

Among them, the subscripts *i* and *t* represent the region and the year, respectively, *v*_*i*_ represents the individual fixation effect, *ε*_*it*_ represents the error terms, GECM represents the green economic efficiency, FDI represents the foreign direct investment, IN represents the regional innovation, SECD represents the secondary industry added value, *RD* represents the R&D spending, and GGPAY represents the fiscal spending. Considering the “inertia” of economic development, the lag phase of green economic efficiency is added to the model. To solve the endogenous problem of introducing lag caused by interpreted variables, its lag term is taken as tool variables.

#### 4.1.3. The Mediation Effect Model

Using Wen et al. [24] for reference, regional innovation is taken as a mediating variable. The model is set as follows:

(12) $$\begin{array}{c} Ln{\text{GECM}}_{it}=\beta_{0}+\beta_{1}Ln{\text{FDI}}_{it}+\sum_{j}\beta_{j}Ln{\text{Control}}_{it}+v_{i}+\varepsilon_{it}, \end{array}$$

(13) $$\begin{array}{c} Ln{\text{IN}}_{it}=\beta_{0}+\lambda_{1}Ln{\text{FDI}}_{it}+\sum_{j-1}\beta_{j-1}Ln{\text{Control}}_{it}+v_{i}+\varepsilon_{it}, \end{array}$$

(14) $$\begin{array}{c} Ln{\text{GECM}}_{it}=\beta_{0}+\lambda_{2}Ln{\text{FDI}}_{it}+\alpha Ln{\text{IN}}_{it}+\sum_{j-1}\beta_{j-1}Ln{\text{Control}}_{it}+v_{i}+\varepsilon_{it}. \end{array}$$

Among them, the subscripts *i* and *t* represent the region and the year, respectively, *v*_*i*_ represents the individual fixation effect, *ε*_*it*_ indicates error terms, GECM represents green economic efficiency, FDI represents foreign direct investment, IN represents regional innovation, and Control represents control variables.

#### 4.1.4. The Dynamic Panel Threshold Model

In order to study whether FDI has a heterogeneity impact on green economic efficiency due to the change of economic development level, the dynamic panel threshold model proposed by Caner and Hansen is used for the empirical test [25]. The advantage is the assumption that explanatory variables are strictly exogenous, considering the endogenous and individual fixation. The model is set as follows:

(15) $$\begin{array}{c} Ln{\text{GECM}}_{it}=\alpha +\beta_{2}Ln{\text{FDI}}_{it}I\left(Ln{\text{GDP}}_{it}<\lambda_{1}\right)+\beta_{3}Ln{\text{FDI}}_{it}I\left(\lambda_{1}\leq Ln{\text{GDP}}_{it}\leq \lambda_{2}\right)\\ +\beta_{4}Ln{\text{FDI}}_{it}I\left(Ln{\text{GDP}}_{it}>\lambda_{2}\right)+\beta_{5}Ln{\text{Control}}_{it}+v_{i}+\varepsilon_{it}. \end{array}$$

Among them, the subscripts *i* and *t* represent the region and the year, respectively, *v*_*i*_ represents the individual fixation effect, *ε*_*it*_ represents the error term, *λ* represents the threshold value, and *Ln*GDP is the pair value of the regional actual GDP and the threshold variable. Control represents the control variable, and *Ln*FDI represents the pair value of the actual amount of foreign capital. The problem related to error term sequence in individual effect elimination (15) uses forward orthogonal discrepancy transform method [26]. We converted formula (15) to

(16) $$\begin{array}{c} Ln{\text{GECM}}^{*}{}_{it}=\alpha +\beta_{2}Ln{\text{FDI}}^{*}{}_{it}I\left(Ln{\text{GDP}}_{it}<\lambda_{1}\right)+\beta_{3}Ln{\text{FDI}}^{*}{}_{it}I\left(\lambda_{1}\leq LnG\;DP_{it}\leq \lambda_{2}\right)\\ +\beta_{4}Ln{\text{FDI}}^{*}{}_{it}I\left(Ln{\text{GDP}}_{it}>\lambda_{2}\right)+\beta_{5}Ln{\text{Control}}_{it}^{*}+v^{*}{}_{i}+\varepsilon^{*}{}_{it}. \end{array}$$

The fitting value of *Ln*GECM^*∗*^_*it*_ is calculated and then substituted into (15) to obtain the threshold fitting value. Finally, the threshold effect is verified based on the threshold fitting value.

### 4.2. Description of the Variables

#### 4.2.1. Variable Selection for the Three-Stage DEA Model

Expected output is measured by actual GDP. Unexpected output is borrowed from Yang and Hu [27]. Using the method, the five pollutants are as follows: industrial wastewater discharge, industrial sulfur dioxide emission, smoke (powder) dust emission, industrial solid waste production, and nitrogen oxide emission. The entropy method of the previously mentioned five pollutants is used to build a comprehensive index of environmental pollution, as the nonexpected output. The input variables are divided into labor input, capital input, and energy investment, respectively, measured by the total number of three industrial employees at the end of the year, capital stock, and energy consumption [28]. The capital stock data of each province over the years are calculated by the perpetual inventory method [29]. The selection basis of environmental variables is able to affect the economy and pass the LR test [30]. The comprehensive empirical test results are measured by the urbanization rate and the number of patent applications^①^.

#### 4.2.2. Variable Selection of Dynamic System GMM and Dynamic Threshold Model

The interpreted variable is the green economic efficiency (GECM_*it*_), based on production efficiency. Consider the quality and quantity of economic growth and measure the relationship between input, expected output, and nonexpected output in production activities. The core interpretation variable is foreign direct investment (FDI_*it*_), measured by the actual amount of foreign investment. Regional innovation (INit) is measured by the number of patent applications. The control variable contains the financial expenditure (GGPAY_*it*_), measured by the total fiscal expenditure. The value of secondary industry (SECDit) is measured by the added value of the secondary industry. R&D expenditure (RDit) is measured by R&D expenditure. Green economic efficiency lags behind phase 1 (GECM_*it−*1_), measured by lagging efficiency of green economy. The threshold variable is the level of economic development (GDP_*it*_), measured by the actual GDP value.

For descriptive data statistics, as shown in Table 2, logarithms of measurement model variants are taken to reduce the effect of heterovariance. The data comes from China Statistical Yearbook, China Environmental Statistical Yearbook, the provincial Statistical Yearbook, and the National Bureau of Statistics. Due to the change of some pollutant statistical caliber and project, occurring in 2017, the study sample period was selected from 2010–2017. Data from Taiwan and Tibet is missing, so they were not included in the investigation scope.

## 5. Empirical Test and Analysis

### 5.1. Results and Analysis of Green Economic Efficiency

Table 1 and Figure 1 show the efficiency value of green economy in China.

Table 1 shows that the mean green economic efficiency of 1 and above are Hainan, Beijing, Jiangsu, and Guangdong, respectively, and the mean green economic efficiency is 1.375, 1.067, 1.085, and 1.000, respectively. The mean green economic efficiency in the bottom provinces are Henan and Shanxi, and the mean green economic efficiency is 0.616 and 0.602 respectively. The samples are further divided into eastern, central, and western regions, and significant regional differences are found compared with the mean regional green economic efficiency (Figure 1). The national average green efficiency of the economy is between 0.810 and 0.850, showing the overall trend of stable and rising. According to the subregional comparison, the average efficiency of eastern green economy is the largest, between 0.888 and 0.936, and is located above the national average level of green economy efficiency. The efficiency value of green economy in western China is between 0.773 and 0.895. Before 2012, the green economy efficiency level of the western region was lower than the national average. After 2012, the efficiency level of green economy was higher than the national average and showed a stable trend. The green economic efficiency value of the central region is between 0.690 and 0.745, indicating that the green economic efficiency in the central region has great potential for improvement.

### 5.2. Benchmark Regression Test and Analysis

To verify the impact of FDI on the green economic efficiency, the dynamic system GMM model is used for empirical tests, as shown in Table 3. From the test results, the *P* value of the AR(2) estimation coefficient is greater than 0.05, indicating that there is no second order autocorrelations in the residual sequence. The *P* value of the Hansen statistics is greater than 0.05, accepting the original assumption that the tool variable is reasonably valid. The estimation coefficients of *Ln*GECM_*it−*1_ are all less than the estimation coefficient of the lag term in column 1 that has the mixed regression results and greater than the lag term estimation coefficient in column 2 that has the fixed effect results, indicating that the GMM estimation results are robust and effective.

From columns 3 to 5 in Table 3, the following is concluded. The coefficient of *Ln*GECM_*it−*1_ is significantly positive, indicating that the efficiency of China's early green economic efficiency is sustainable and significantly positively promoting the green economic efficiency in the future. The coefficient of *Ln*SECD_*it*_ is robust and significantly negative, indicating that the secondary industry plays a negative role on green economic efficiency. The reason is that the nonexpected output mostly comes from the secondary industry. The secondary industry leads to the excessive increase of pollutant emissions while promoting economic growth, which is not conducive to the green development of economy. Add the *Ln*FDI_*it*_, *Ln*IN_*it*_ in the columns 3 and 4, respectively, and add both *Ln*FDI_*it*_ and *Ln*IN_*it*_ items to column 5 for verification. It can be found that the regression coefficient of *Ln*FDI_*it*_ is always significantly positive, indicating that FDI can significantly promote the improvement of the efficiency of green economy, which partially confirms the “pollution halo” hypothesis. Meanwhile, the estimation coefficient of *Ln*IN_*it*_ is always significantly positive, suggesting that regional innovation can also promote growth in green economic efficiency. The reasons are as follows. First, the number of patent applications is the embodiment of high-tech innovation achievements, which can directly improve production efficiency and achieve the growth of industrial competitiveness, which plays an important and positive role in the economy. Second is the innovation-driven development. The wide application of high-tech can drive the transformation of industrial structure from low level to high level, enhance the correlation effect between industries, and promote the harmless treatment of waste generated in production activities, so as to realize the green development of economic economy. In conclusion, the test results verify hypothesis 1 of this paper.

### 5.3. Regional Heterogeneity Test and Analysis

It has been verified that FDI has a positive impact on China's overall green economic efficiency. This section divides China into eastern, central, and western regions to further examine the possible heterogeneity impact of FDI on the green economic efficiency of the east, center, and west. The empirical results are shown in Table 4. Both the AR(2) and Hansen tests have passed the test, so the empirical results are robust and effective.

According to the test results of columns 1 and 2 in Table 4, the estimated coefficient of *Ln*FDI_*it*_ in the eastern region was 0.0345 and passed the significance level test of 10%, while the estimated coefficient of *Ln*FDI_*it*_ in the central region was 0.1441 and passed the significance level test of 1%. According to column 3, the estimated coefficient of *Ln*FDI_*it*_ in the western region is 0.0342, but it fails to pass the significance test. It can be seen that FDI has a positive and significant promoting effect on the green economic efficiency in the eastern and central regions of China, while the positive effect on the green economic efficiency in the western regions is not significant, indicating that FDI's promoting effect on the green economic efficiency has significant regional heterogeneity. Further investigation of the number of FDI, patent applications, and industrial structure in the eastern, central, and western regions shows that the average value of FDI in the eastern region is 84 billion yuan, the average number of patent applications is 137249, and the average value added of the secondary industry is 14790 billion yuan. In the central region, the average FDI was 443 billion yuan, the average number of patent applications was 41508, and the average value added of the secondary industry was 10334 billion yuan. In the western region, the average FDI was 139 billion yuan, the average number of patent applications was 28998, and the average value added of the secondary industry was 5247 billion yuan. In the comprehensive analysis, the reasons for the regional heterogeneity impact of FDI on green economy efficiency are as follows. First of all, the economic development level in the eastern and central regions is higher, the industry sector development is relatively perfect, and the transformation of science and technology ability is strong, which is able to advance the experience of the foreign side and introduce high and new technology to efficiently absorb transformation, promote regional technology progress, improve the utilization ratio of capital, and better achieve the efficiency of the green economy growth. Second, the number of foreign capital in the eastern and central regions is relatively sufficient. Due to the limitation of geographical location and the small stock of FDI in the western region, it is difficult to produce an effective capital accumulation. Meanwhile, the estimated coefficient of *Ln*IN_*it*_ in the eastern region is significantly positive, while the central and western regions are not significant as a whole, indicating that the innovation in the eastern region has a stronger role in promoting the efficiency of green economy.

## 6. Empirical Test of Influence Mechanism

### 6.1. Mediating Effect Test and Analysis

The test results are shown in Table 5. It can be seen from column 1 that the regression coefficient of *Ln*FDI_i*t*_ is 0.0669 and has passed the 1% significance test. From column 2, the regression coefficient of *Ln*FDI_*it*_ is 0.3037 and has passed the 1% significance test. The results indicate that FDI has a significant positive promotion effect on regional innovation. From column 3, the regression coefficient of *Ln*IN_*it*_ is 0.0394 and has passed the 10% significance level test, indicating that the mediating effect of regional innovation is significant. The reasons are as follows. On the one hand, the technology spillover effect of FDI promotes the scientific and technological innovation research and development among industries through capital flow, personnel factor flow, and technology exchange and promotes the popularization of high and new technologies, so as to realize the positive promotion of green economic efficiency. On the other hand, FDI into the domestic market will cause competition effect and demonstration effect, especially for domestic high-tech enterprises, advanced production technology to squeeze domestic enterprises, forcing domestic high-tech enterprises to imitate foreign enterprises to increase the independent scientific research and innovation experiment and improve independent innovation ability, so as to promote the technological progress of the whole region [31]. Finally, it can be seen from column 1 that the regression coefficient of *Ln*FDI_*it*_ is significant and from column 3 that the regression coefficient of both *Ln*FDI_*it*_ and *Ln*IN_*it*_ is significantly positive, which verifies the significance and robustness of the mediation effect. In conclusion, the test results verify hypothesis 2 of this paper.

### 6.2. Threshold Effect Test and Analysis

To further verify whether the impact of FDI on green economy efficiency changes with the level of economic development, this section will build a dynamic panel threshold model for empirical testing.

Repeat 400 calculation threshold, *F* inspection, and confidence interval by self-inspection method, and the results are shown in Table 6. It is seen from Table 6 that both the single threshold value and the double threshold values are significant, and the three threshold values do not pass the significance test. The single threshold is included in the double threshold. In order to ensure the validity of the threshold value, the threshold value is tested, and the likelihood ratio test results (Figure 2) can know that the double threshold values are valid, so the double panel threshold model is selected.

The test results are shown in Table 7. According to the threshold value, it is seen from Table 7 that when the threshold is less than 8.748, the estimated coefficient of FDI is −0.0554 and has passed the 1% significance level test, indicating that FDI has a negative impact on green economic efficiency. When the threshold is between 8.748 and 9.373, the estimated coefficient of FDI is 0.0347, failing the significance test. When the threshold is greater than 9.373, the estimated coefficient of FDI is 0.0628 and has passed the 1% significance level test, indicating that FDI can positively promote green economic efficiency. Further comparison of the interval regression samples shows that the western region occupied the vast majority of the samples where the economic level was under the first threshold. The samples between the double thresholds are samples of the western and central regions, mainly, Shanxi, Inner Mongolia, Jilin, Heilongjiang, Guizhou, Yunnan, Shaanxi, Gansu, and Xinjiang. The sample above the second threshold contains the entire eastern, a few central, and a very few western regions. In addition, compared with the number of foreign investment, the number of patent applications, and the second output value of different sections, it is seen that, in the areas with the economic level below the first threshold, the corresponding average number of foreign investment is 37 billion yuan, the average number of patent applications is 3771, and the average output value of the secondary industry is 1455 billion yuan. When economic level is between the double thresholds, the average number of foreign capital is 144 billion yuan, the average patent applications is 15659, and the average output value of the secondary industry is 4705 billion yuan. For areas with economic level higher than the second threshold, the corresponding average number of foreign capital is 689 billion yuan, the average number of patent applications is 104269, and the average output value of the secondary industry is 13751 billion yuan. In conclusion, regions with economic level higher than the second threshold value have more sufficient scale of foreign capital and stronger regional innovation ability. It can be inferred that the heterogeneity impact of FDI on green economic efficiency at different economic levels is as follows. First, the insufficient number of FDI in the middle and lower reaches of the economic level leads to the insignificant promotion effect of FDI capital accumulation effect. Second, the demonstration and guiding role of foreign investment in the middle and downstream economic areas is weak. There are few high-tech talents in these areas and the production technology is relatively backward, so the technology spillover cannot absorb and transform foreign investment in a timely and effective manner. To sum up, the test results verify hypothesis 3 of this paper.

### 6.3. Test of Robustness

To further test the robustness of the threshold results, this paper draws on the robustness test method of Li et al. [32]. The panel threshold model is similar in a sense to adding virtual variables, which is structurally similar to the cross term model, where the panel threshold model can get exactly the structural change point and the cross term cannot. The model set below is to assume the nonlinear influence of FDI on green economic efficiency and then introduce the quadratic term of FDI, set as follows:

(17) $$\begin{array}{c} Ln{\text{GECM}}_{it}=\alpha +\beta_{2}{\text{FDI}}_{it}^{2}*Ln{\text{FDI}}_{it}+\beta_{3}{\text{FDI}}_{it}*Ln{\text{FDI}}_{it}+\beta_{4}Ln{\text{Control}}_{it}+v_{i}+\varepsilon_{it}. \end{array}$$

In (17), the meaning of each variable remains unchanged from the previous one in this paper, and the marginal effect of *Ln*FDI_*it*_ on *Ln*GECM_*it*_ can be obtained:

(18) $$\begin{array}{c} \frac{\partial L\;n{\text{GECM}}_{it}}{\partial L\;n{\text{FDI}}_{it}}=\beta_{2}{\text{FDI}}_{it}^{2}+\beta_{3}{\text{FDI}}_{it}. \end{array}$$

In conclusion, if *β*_*2*_ and *β*_*3*_ can pass the significance test, it is verified that there is a nonlinear relationship between the effect of FDI on green economic efficiency.

The test results are shown in Table 8, and the test results show that the GMM estimation result of the cross model is reasonable and effective [33]. First, both the quadratic and primary term coefficients in the model are significant, confirming the nonlinear relationship between FDI and the green economic efficiency and further confirming the robustness of the threshold effect results [34].

## 7. Research Conclusions and Policy Implications

At the time of the transformation of China's old drivers of economic growth, improving the level of foreign investment and domestic economic allocation is an important direction for improving the level of participation in the international cycle and an important link in the process of building a new pattern of development, in which domestic and international cycles mutually promote. Based on the basis of existing research results, the influence mechanism of FDI, and regional innovation on green economic efficiency, we calculated the basis of 30 provincial-level panel data from 2010 to 2017, tested the driving effect of FDI, regional innovation on green economic efficiency, and tested the driving status of FDI on green economic efficiency by regions. On this basis, the intermediary effect model is constructed to test the influence mechanism of regional innovation as the intermediary variable on this driving action. The dynamic panel threshold model was used to examine the influence of FDI on green economic efficiency under different levels of economic development. The main research conclusions are as follows: (1) FDI has a significant driving effect on green economic efficiency. Further regional heterogeneity analysis found that FDI has a significant positive driving effect on green economic efficiency in the eastern and central regions, and the driving effect in the western region is not significant. (2) The analysis of the influence mechanism has found that the role path of regional innovation is significantly positive, and FDI can improve the efficiency of green economy by promoting regional innovation. FDI has a significant effective double threshold for the level of economic development. When the economic level is below the first threshold value, FDI promotes the green economic efficiency between the first threshold value and the second threshold value; when the economic level crosses the second threshold value, FDI has a significant positive effect on the green economic efficiency [35].

Based on the previously mentioned conclusions, this paper puts forward the following two policy inspirations. (1) At present, China should increase the policy support for introducing foreign investment in backward regions and coordinate the reasonable allocation of foreign investment in various regions. At present, there are great differences in the amount of foreign investment in various provinces and cities. In order to promote the rational allocation of foreign capital and further promote regional coordination and green development, the government should adjust the introduction policy and intensity of foreign investment on the basis of opening up, combined with the characteristics of regional distribution and the level of economic development. For provinces and cities with low economic level, the government needs to formulate more attractive and biased policies to attract foreign capital and at the same time improve the supporting facilities of regional economic development, realize the improvement of regional comprehensive economic strength, make foreign capital attract, stay, and live for a long time, and strengthen the positive effect of the green economic efficiency of the region. For provinces and cities with high economical level, the government's investment policy needs to take dimension and stability as the main goal, and stabilize the introduction of foreign investment to continue to play the role of FDI in promoting the green economic efficiency. (2) The regional innovation and the transformation of original achievements should be encouraged. From the perspective of regional innovation, innovation is conducive to the improvement of green economy efficiency, and FDI can improve the efficiency level of green economy by promoting regional innovation. The government should improve the support of new technology and new knowledge innovation policy, strengthen the pertinence and support of regional foreign investment, solve the shortage of enterprise research and development funds, high and new technology efficiency, and achievement transformation difficulties, realize science and technology from “follow” to “and run” to the hierarchy of “leading” change, and further strengthen the FDI and regional innovation promoting green economic efficiency.

## 8. Research Deficiencies and Prospects

1. This paper measures the impact of FDI capital on China's green economic efficiency from the perspective of factor input and uses the three-stage DEA model to put forward the impact of environmental factors, statistical factors, and other factors, which is a relatively cutting-edge exploration. Due to the particularity of research perspective and level, the continuity and timeliness of environmental pollutant data published in relevant databases are limited, which makes it difficult to timely and comprehensively reveal the recent changes of FDI on China's green economy efficiency. After the database update data and the statistical classification of core industries of digital economy are officially published in the future, more samples and perspectives can be used for empirical testing from a more accurate digital industry classification.
2. Green economic efficiency has rich practical connotation. This paper makes a preliminary exploration from the threshold effect model and intermediary effect model by using the provincial panel data. The follow-up research can also start from the municipal panel data and use the spatial econometric model to verify the spatial spillover effect of FDI on green economic efficiency from the perspective of spatial correlation and explore whether there is a “club agglomeration phenomenon” between FDI and green economic efficiency in space, so as to enrich the perspective of the impact of FDI on green economic efficiency.

## Figures and Tables

**Figure 1:** Green economic efficiency trend.

**Figure 2:** The LR test results of the double threshold values.

**Table 1:** Green economic efficiency.

DMU	2010	2014	2017	Mean
Beijing	1.058	1.005	1.107	1.067
Tianjin	0.688	0.723	1.027	0.772
Hebei province	0.640	0.666	0.611	0.651
Shanxi province	0.604	0.619	0.550	0.602
Inner Mongolia	0.674	0.693	0.625	0.688
Liaoning province	0.696	0.705	0.646	0.694
Jilin province	0.671	0.753	0.704	0.723
Heilongjiang province	0.689	0.729	0.682	0.713
Shanghai	1.045	0.887	1.074	0.973
Jiangsu province	1.065	1.104	1.085	1.085
Zhejiang province	0.929	0.948	0.897	0.925
Anhui province	0.707	0.781	0.733	0.763
Fujian province	0.876	0.844	0.802	0.870
Jiangxi province	0.863	0.870	0.822	0.904
Shandong province	0.731	0.774	0.755	0.754
Henan province	0.600	0.636	0.598	0.616
Hubei province	0.734	0.763	0.746	0.747
Hunan province	0.712	0.765	0.754	0.741
Guangdong province	1.000	1.000	1.000	1.000
Guangxi province	1.179	0.707	0.614	0.764
Hainan province	1.328	1.289	1.420	1.375
Chongqing	0.738	0.811	0.870	0.794
Sichuan province	0.639	0.732	0.718	0.700
Guizhou province	0.656	1.039	1.075	0.907
Yunnan province	0.566	0.651	0.687	0.652
Shaanxi province	0.687	0.921	0.805	0.848
Gansu province	0.716	1.007	0.963	0.965
Qinghai province	1.157	1.213	1.236	1.211
Ningxia province	1.017	0.872	0.845	0.906
Xinjiang province	0.778	0.767	0.671	0.751

Due to space limitation, only green economic efficiency of some years was included.

**Table 2:** Variable descriptive statistics.

Variables	Number of observations	Minimum value	Maximum value	Mean	Standard deviation
Expected output	240	1350.43	79976.42	20571.87	—
Unexpected output	240	6455.64	220000.00	57595.17	—
	240	307.65	6767.00	2735.28	—

Investment variable	240	10579.00	250000.00	81306.36	—
	240	1358.51	38899.25	14551.74	—

Urbanization rate	240	33.81	89.60	55.93	—
Number of patent applications	240	602.00	627834.00	76051.88	—
*Ln*GECM_*it*_	240	−0.23	0.52	≤0.001	0.10
*Ln*FDI_*it*_	240	−0.04	7.74	5.43	1.65
*Ln*IN_*it*_	240	6.40	13.35	10.37	1.46
*Ln*GGPAY_*it*_	240	6.32	9.62	8.18	0.59
*Ln*SECD_*it*_	240	6.35	10.59	8.92	0.92
*Ln*RD_*it*_	240	10.96	16.76	14.13	1.33
*Ln*GDP_*it*_	240	9.63	0.85	7.21	11.29

**Table 3:** Benchmark regression test.

Variables	PLS	PLS_FE	GMM	GMM	GMM
	1	2	3	4	5
*Ln*GECM_*it*−1_	0.8749^*∗∗∗*^	0.3441^*∗∗∗*^	0.6892^*∗∗∗*^	0.6340^*∗∗∗*^	0.5170^*∗∗∗*^
	[29.68]	[5.57]	[7.36]	[5.16]	[5.16]

*Ln*FDI_*it*_	0.0029	−0.0075	0.0669^*∗∗∗*^	—	0.0587^*∗∗*^
	[0.58]	[−0.60]	[3.06]	—	[2.38]

*Ln*IN_*it*_	0.0227^*∗∗∗*^	−0.0531^*∗∗*^	—	0.0507^*∗∗∗*^	0.0394^*∗*^
	[2.60]	[−2.00]	—	[3.78]	[1.73]

*Ln*SECD_*it*_	−0.0478^*∗∗∗*^	0.1285	−0.1456^*∗∗∗*^	−0.1019^*∗∗∗*^	−0.1792^*∗∗∗*^
	[−3.06]	[1.38]	[−3.74]	[−3.11]	[−4.24]

*Ln*RD_*it*_	0.0034	0.0011	0.0006	0.0014	−0.0001
	[0.94]	[0.32]	[0.11]	[0.34]	[−0.03]

*Ln*GGPAY_*it*_	−0.0033	−0.0064	0.0472	−0.0026	0.0253
	[−0.15]	[−0.10]	[1.18]	[−0.07]	[0.57]

CONS	0.1334	−0.6437	0.4876^*∗∗*^	0.324	0.5823^*∗∗*^
	[1.08]	[−1.62]	[2.25]	[1.56]	[2.41]

AR(2)	—	—	0.2100	−0.3000	−0.0700
	—	—	(0.834)	(0.766)	(0.945)

Hansen	—	—	25.7700	24.5500	23.7100
	—	—	(0.174)	(0.219)	(0.208)

Individual effects	—	Control	Control	Control	Control

*F*	266.0000	8.4900	30.4900	53.2800	28.6400
	(≤0.001)	(≤0.001)	(≤0.001)	(≤0.001)	(≤0.001)

(1) The values in are *t* statistical value of regression coefficient in the same table below; the values in () are *P* value of corresponding test statistics in the same table below; (2) ^*∗∗∗*^, ^*∗∗*^, and ^*∗*^ indicate significant significance at 1%, 5%, and 10%, respectively. All tables are the same.

**Table 4:** Empirical test of regional heterogeneity.

Interpretation variables	East	Center	West
	1	2	3
*Ln*GECM_*it*−1_	0.6397^*∗∗∗*^	0.5934^*∗∗∗*^	0.9231
	[3.19]	[4.28]	[1.28]

*Ln*FDI_*it*_	0.0345^*∗*^	0.1411^*∗∗∗*^	0.0342
	[2.10]	[3.51]	[0.20]

*Ln*IN_*it*_	0.0362^*∗*^	−0.0175	0.0443
	[2.07]	[−1.23]	[0.22]

*Ln*SECD_*it*_	−0.0852^*∗∗*^	0.0024	−0.1450
	[−2.46]	[0.02]	[−0.40]

*Ln*RD_*it*_	−0.0011	−0.0136^*∗*^	−0.0192
	[−0.14]	[−2.07]	[−0.25]

*Ln*GGPAY_*it*_	0.0028	−0.3051^*∗*^	−0.0414
	[0.10]	[−2.09]	[−0.09]

CONS	0.1084	1.9121^*∗∗∗*^	1.2626
	(0.011)	[3.39]	[0.25]

AR(2)	−0.7100	−0.3800	0.7400
	(0.480)	(0.703)	(0.460)

Hansen	6.6000	3.0400	4.2600
	(0.999)	(0.386)	(1.000)

Individual effects	Control	Control	Control

*F*	57.8200	12.2600	5.6600
	(0.000)	(0.001)	(0.019)

**Table 5:** Empirical test of the mediating effect.

Variables	1	2	3
	*Ln*GECM_*it*_	*Ln*IN_*it*_	*Ln*GECM_*it*_
*Ln*FDI_*it*_	0.0669^*∗∗∗*^	0.3037^*∗∗∗*^	0.0587^*∗∗*^
	[3.06]	[4.34]	[2.38]

*Ln*IN_*it*_	—	—	0.0394^*∗*^
	—	—	[1.73]

*Ln*GECM_*it*−1_	0.6892^*∗∗∗*^	1.1262	0.5170^*∗∗∗*^
	[7.36]	[1.48]	[5.16]

*Ln*SECD_*it*_	−0.1456^*∗∗∗*^	0.4393^*∗*^	−0.1792^*∗∗∗*^
	[−3.74]	[1.92]	[−4.24]

*Ln*GGPAY_*it*_	0.0472	1.0455^*∗∗∗*^	0.0253
	[1.18]	[3.24]	[0.57]

*Ln*RD_*it*_	0.0006	0.0071	−0.0001
	[0.11]	[0.38]	[−0.03]

*CONS*	0.4876^*∗∗*^	−3.6150^*∗∗*^	0.5823^*∗∗*^
	[2.25]	[−2.72]	[2.41]

AR(2)	0.2100	0.7400	−0.0700
	(0.834)	(0.461)	(0.945)

Hansen	25.7700	22.5500	23.7100
	(0.174)	(0.258)	(0.208)

Individual effects	Control	Control	Control

*F*	30.4900	92.0100	28.6400
	(0.000)	(0.000)	(0.000)

**Table 6:** The threshold value estimation and test.

The threshold is set up variables	Number of thresholds	Threshold	The *F* value	10%	5%	1%	The 95% confidence interval
*Ln*GDP_*it*_	Single	8.748	42.9450^*∗∗∗*^	8.484	15.724	32.288	[8.748,8.819]
	Double	8.748; 9.373	20.2960^*∗∗∗*^	3.474	4.628	7.604	[8.748,8.819]; [9.250,9.373]
	Three	9.118	0.0000	0.000	0.000	0.000	[9.027,9.124]

**Table 7:** Empirical test of the threshold effect.

Variables	1	2	3
Threshold variable	*Ln*GDP_*it*_ < 8.748	8.748 ≤ LnGDP_*it*_ ≤ 9.373	*Ln*GDP_*it*_ > 9.373

*Ln*FDI_*it*_	*Ln*GDP_*it*_ < 8.748	8.748 ≤ *Ln*GDP_*it*_ ≤ 9.373	*Ln*GDP_*it*_ > 9.373
	−0.0554^*∗∗∗*^	0.0347	0.0628^*∗∗∗*^

*Ln*GECM_*it*−1_	[−2.97]	[0.60]	[5.67]
	0.3135^*∗∗∗*^	0.1832	0.3468^*∗∗∗*^

Control variable	[2.80]	[0.27]	[7.54]
Individual effects	Control	Control	Control

Sargan	Yes	Yes	Yes
	19.7496	1.1150	16.1430

AR(2)	(0.474)	(1.000)	(0.933)
	—	1.2718	0.0453

Wald	—	(0.203)	(0.964)
	201.6500	59.0700	2058.8500

When the *Ln*GDP_*it*_ < 8.748, since the two-step estimator variance-covariance matrix is not full rank, the one-step estimation is taken, and the results are still robust and without the AR(2) test.

**Table 8:** Robustness test results.

Variables	GMM	Variables	GMM
*Ln*GECM_*it−1*_	0.4157^*∗∗*^	AR(2)	−0.5900
	[2.07]		(0.554)

FDI_*it*_^2^*∗Ln*FDI_*it*_	−5.67e−08^*∗*^	Hansen	21.1100
	[−1.71]		(0.133)

FDI_*it*_*∗Ln*FDI_*it*_	0.0001^*∗*^	*F*	9.5300
	[1.91]		(≤0.001)

Control variable	Control	—	—

## Data Availability

The data used to support the findings of this study are included within the article.
